# Doppler Echocardiography Combined with NTproBNP/BNP in the Diagnosis of Pulmonary Artery Hypertension Associated with Congenital Heart Disease

**DOI:** 10.1155/2023/1896026

**Published:** 2023-02-13

**Authors:** Xi Zhang, Zhinan Zhai, Xu Geng, Yanbo Zhu, Shijuan Yang, Tongyun Chen, Xue Wu, Jingkun Zhang, Zhi-Gang Guo, Min Hou

**Affiliations:** ^1^Department of Clinical Laboratory, Clinical School of Thoracic, Tianjin Medical University, Tianjin 300222, China; ^2^Department of Clinical Laboratory, Tianjin Chest Hospital, Nankai University, Tianjin 300222, China; ^3^Department of Clinical Laboratory, Chest Hospital, Tianjin University, Tianjin 300222, China; ^4^Department of Ultrasonography, Tianjin Chest Hospital, Tianjin 300222, China; ^5^Department of Cardiovascular Surgery, Tianjin Chest Hospital, Tianjin 300222, China; ^6^Institute for Global Health Sciences, University of California, San Francisco, CA, USA; ^7^Cardiovascular Research Institute, University of California, San Francisco, CA, USA

## Abstract

**Background:**

Pulmonary artery hypertension (PAH) is a common complication of congenital heart disease (CHD) and is associated with worse outcomes and increased mortality. The Doppler echocardiography (DE) is a commonly used imaging tool for both diagnosis and follow-up examination of PAH. Here is to evaluate the diagnostic performance of DE combined with NTproBNP/BNP as screening strategy in PAH patients with CHD.

**Methods:**

A retrospective study in 64 patients with CHD has been carried out to compare estimate pulmonary artery systolic pressure (PASP) measured with DE to that measured with right heart catheterization (RHC). The Pearson correlation analyses were used to calculate the correlation coefficients between RHC and DE. The Bland-Altman analyses were carried out to assess the agreement between the two methods. ROC analyses were used to evaluate the diagnostic performance of DE, NTproBNP/BNP, and DE combined with NTproBNP/BNP.

**Results:**

Our data have demonstrated that a mild correlation (*r* = 0.4401, *P* < 0.01) was observed between PASP (78.1 ± 29.0 mmHg) measured during RHC and PASP (74.9 ± 19.7 mmHg) as estimated using DE. The Bland-Altman analysis demonstrated that the bias for DE PASP estimates was 3.2 mmHg with 95% limits of agreement ranging from -49.53 to 55.90 mmHg. The results of DE showed an AUC of 0.848 (95% CI = 0.666-1; *P* < 0.001), the sensitivity of which was 98.3% and the specificity was 77.8%. The AUC of NTproBNP/BNP for the identification of PAH was 0.804 (95% CI = 0.651-0.956; *P* < 0.001), the sensitivity of which was 81.4% and the specificity was 87.5%. The AUC of DE combined with NTproBNP/BNP was 0.857 (95% CI = 0.676-1; *P* < 0.001), of which sensitivity was 100% and specificity was 77.8%. The positive predictive value (PPV) and negative predictive value (NPV) were 96.6% and 100%, respectively.

**Conclusions:**

Our study shows that the Doppler echocardiography combined with NTproBNP/BNP has better diagnostic performance in pulmonary artery hypertension associated with congenital heart disease, especially when DE negative screening in PAH patients.

## 1. Introduction

Congenital heart disease, referred to as CHD, is an abnormality of cardiovascular morphology, structure, and function caused by developmental disorders of the heart and blood vessels, with an incidence of about 7‰ to 10‰ in live births, and is the primary birth defect disease in humans. In adults, approximately 6.5%-10% of CHD patients will develop into pulmonary artery hypertension (PAH) [1]. The assessment of PAH directly affected the timing of CHD surgery, surgical methods, and prognosis. However, right heart catheter (RHC) is an invasive examination with high risk, requiring professional equipment as well as experienced physicians, especially low birth weight newborns have poor tolerance to RHC, while the Doppler echocardiography (DE) is widely used for its simplicity, cheapness, and ease. Pulmonary arterial systolic pressure (PASP) is considered close to right ventricular systolic pressure (RVSP) in the exclusion of right ventricular outflow tract obstruction [2].

NTproBNP or BNP are secreted by cardiomyocytes due to excessive stretching of the ventricles, which remain the most promising blood biomarkers for risk prediction of patients with PAH [3].

Here, we investigate the accuracy of DE and, further, DE combined with NTproBNP/BNP in estimating the pulmonary arterial pressure of patients with CHD by comparing with RHC.

## 2. Methods

### 2.1. Study Population

A total of 64 patients diagnosed as CHD or PAH associated with congenital heart disease (PAH-CHD) by the Doppler echocardiography (DE) and RHC who were hospitalized in the Department of Cardiovascular Surgery, Tianjin Chest Hospital, between March 2017 and March 2022 were collected. All patients had no right ventricular outflow tract obstruction and tricuspid valve prolapse and no family history of pulmonary hypertension. The RHC examination was performed within 72 h after the DE examination, and the relevant parameters were recorded. This study was approved by the Ethics Committee of Tianjin Chest Hospital, and all patients and their families signed informed consent.

### 2.2. Evaluation Criteria for PAH

The 2015 European Society of Cardiology/European Respiratory Society (ESC/ERS) guidelines for the diagnosis and treatment of pulmonary hypertension was used: mean pulmonary arterial pressure ≥ 25 mmHg by right heart catheterization at sea level and at rest [4]. Furthermore, according to the 2015 Chinese Expert Consensus on Diagnosis and Treatment of Pulmonary Arterial Hypertension Associated with Congenital Heart Disease, according to the degree of PASP, the patients were divided into as follows: normal PAH: 15-30 mmHg, mild PAH: 31-45 mmHg, moderate PAH: 46-70 mmHg, and severe PAH: > 70 mmHg.

### 2.3. Doppler Echocardiography

Philips IE 33 Doppler ultrasonic diagnostic apparatus was applied with a probe frequency of 1 ~ 5 MHz. Supine position was placed before testing; the tricuspid valve area, tricuspid pressure gradient, left-to-right shunt pressure gradient, right atrial and right ventricular diameters, main pulmonary artery, tricuspid annular systolic excursion, and ejection fraction were measured under two-dimensional ultrasound at the end of expiration. Under the condition of excluding right ventricular outflow tract obstruction, according to the simplified Bernoulli equation, pulmonary artery systolic pressure (PASP = 4*V*max^2^ + right atrial pressure (RAP), where *V* is the maximum velocity of tricuspid valve) was estimated with the tricuspid valve method (hereinafter referred to as the three-back method), and for PDA and VSD cases, PASP (PASP = sBP − 4*V*max^2^, where *V* is the maximum velocity of left-to-right shunt and sBP is the systolic pressure of brachial artery) was also estimated with the left-to-right shunt differential pressure method (hereinafter referred to as the differential pressure method).

### 2.4. Right Heart Catheterization

Standardized right heart catheterization was performed in patients under basic anesthesia, and their pressures were continuously measured: vena cava pressure, right atrial pressure (RAP), pulmonary arterial pressure (PAP), pulmonary arteriolar wedge pressure (PCWP), and aortic pressure; the saturation of each cardiac chamber and great vessels was measured. Hemodynamic parameters such as pulmonary blood flow (Qp), systemic blood flow (Qs), pulmonary circulation resistance (RP), systemic vascular resistance (Rs), and pulmonary vascular resistance (PVR) were calculated by the Fick method.

### 2.5. NTproBNP and BNP Plasma Levels

Blood was collected after admission and transferred immediately to the Department of Laboratory. The samples were processed and analyzed using CLIA assay for plasma BNP (CL-6000i, Mindray, China) and ECLIA assay for serum NTproBNP concentrations (Cobas® e602, Roche, Switzerland). The normal reference range of NTproBNP was 0-300 pg/ml and also 0-100 pg/ml for BNP in our laboratory.

### 2.6. Statistical Analysis

SPSS 22.0 was used for statistical analysis, and *P* < 0.05 was defined as statistically significant difference. Mean ± SD was calculated to present continuous data, while the percent and frequency were used to present categorical data. Chi-square test and Student's *t*-test were used to analyze data when appropriate. Statistical significance was defined as a two-side value of *P* < 0.05. The Pearson correlation analyses were used to calculate the correlation coefficients between RHC and DE.

## 3. Results

### 3.1. Patients' Baseline Characteristics and Hemodynamics

A total of 64 CHD patients were prospectively enrolled in this study. All of the patients estimated PASP using both DE and RHC. Patients' baseline characteristics are presented in Table 1. Sixty-four patients were aged 43.8 ± 18.3 years, and 28.1% were males. The clinical diagnoses of these patients are presented in Table 1: atrial septal defect (57.8%), ventricular septal defect (2.2%), and patent ductus arteriosus (1.8%).

A wide range of PASP (33-160 mmHg by RHC and 25-110 mmHg by DE) was measured. A mild correlation was observed between PASP (78.1 ± 29.0 mmHg) by RHC and PASP (74.9 ± 19.7 mmHg) by DE (*r* = 0.4401, *P* < 0.01) (Figure 1). Using the Bland-Altman analysis, a bias for PASP DE estimates was determined to be 3.2 mmHg with 95% limits of agreement ranging from -49.53 to 55.90 mmHg (Figure 2).

### 3.2. The Diagnostic Performance of DE and DE Combined with NTproBNP/BNP for PAH-CHD

Here, PAH was defined as a PASP ≥ 30 mmHg, pulmonary artery wedge pressure ≤ 15 mmHg, and PVR index > 3 wood units·m^2^ by RHC. And also, PAH was identified when PASP > 40 mmHg or mean PAP ≥ 25 mmHg at rest either by DE. ROC curve analyses were constructed to evaluate the predictive values of DE with/or NTproBNP/BNP levels for the identification of PAH (Figure 3). The results of DE showed an AUC of 0.848 (95% CI = 0.666-1; *P* < 0.001), the sensitivity of which was 98.3% and the specificity was 77.8%. The AUC of NTproBNP/BNP for the identification of PAH was 0.804 (95% CI = 0.651-0.956; *P* < 0.001), the sensitivity of which was 81.4% and the specificity was 87.5%. The AUC of DE combined with NTproBNP/BNP was 0.857 (95% CI = 0.676-1; *P* < 0.001), of which sensitivity was 100% and specificity was 77.8%. The positive predictive value (PPV) and negative predictive value (NPV) are listed in Table 2.

## 4. Discussion

The blood flow of left-to-right shunt in CHD continuously impacts the pulmonary artery, causing vascular remodeling, which in turn leads to the progressive increase of pulmonary arterial pressure and resistance, and finally reverses the blood flow direction to right-to-left and develops into Eisenmenger's syndrome (ES). Therefore, accurate diagnosis, follow-up, and timely intervention of PAH are of great clinical significance. Although the Doppler echocardiography is an excellent noninvasive screening tool for PAH, it has limited accuracy in estimating the right ventricular systolic pressure in PAH and is typically used for assessing the risk of PAH rather than for diagnosis [5]. Many humoral regulators are involved in the regulation of the cardiovascular system during the development of PAH. Circulating BNP and NTproBNP levels have been demonstrated related to PAH: NTproBNP levels correlate with mPAP, PVR, RAP, and cardiac index [6, 7]. An increase of NTproBNP level may reflect right ventricular remodeling leading to impaired right ventricular systolic function [8]. Overall, a correlation was reported that ranged from *r* = 0.31 to *r* = 0.99 [9].

According to Tsujimoto et al.'s review [10], a fixed specificity of 86%, the estimated sensitivity derived from the median value of specificity using HSROC model was 87% in assessing the diagnostic accuracy of the Doppler transthoracic echocardiography for the diagnosis of PAH, which is higher than the specificity (77.8%) in our study (Table 2).

Our study is a retrospective study assessing the value of DE in estimating pulmonary arterial pressure and diagnosing pulmonary hypertension and has a sample size of 64 subjects. We controlled for the time interval between the two examination methods within 72 hours, as well as the parameters measured and the examination conditions. These control measures will greatly reduce the limitations of the study and improve the credibility of the research. In our study, PASP estimated by DE showed a relatively mild correlation in linear regression analysis with PASP by RHC measurements in patients with CHD, and these results were consistent with previous studies [11–13].

Since pathological changes in the pulmonary arteries occur prior to cardiac affection in PAH, pulmonary derived biomarkers would be optimal to detect early PAH. However, although such biomarkers are promising results that have recently been reported as TGF-*β*1 and VEGF165b [14, 15], they are not yet established in clinical use. BNP is a hormone precursor synthesized and released from the atria and ventricles and becomes active BNP and NTproBNP after digestion [16]. BNP reduces blood volume by increasing systemic vascular permeability and natriuretic effects and relaxes vascular smooth muscle cells by increasing intracellular cGMP synthesis, both of which reduce blood pressure and ventricular preload. BNP has a plasma half-life of 22 minutes and NTproBNP is 2 hours. NTproBNP/BNP have been widely used as noninvasive markers and prognostic markers of cardiac dysfunction and are currently the only biomarkers recommended by PAH risk stratification guidelines [17]. Analysis of NTproBNP is available in several laboratories, and the diagnostic cut-off is 300 pg/ml at our laboratory. Here, ROC was used for the diagnosis of PAH by DE and NTproBNP/BNP plasma levels. The AUC of DE combined with NTproBNP/BNP was 0.857, of which sensitivity was 100% and specificity was 77.8%. The positive predictive value (PPV) and negative predictive value (NPV) were 96.6% and 100%, respectively.

The NPV is higher than the single detection, suggesting that, when the Doppler echocardiography fails to detect while PAH is suspected by clinicians, BNP or NT-proBNP are useful as subsequent screening tests.

In summary, our study also showed that the accuracy, sensitivity, specificity, positive predictive value, and negative predictive value of NTproBNP/BNP combined with the Doppler echocardiography for the prognosis prediction of pulmonary hypertension in CHD-PAH patients were higher than those of single detection. The results are consistent with the research of Yin et al. [18], and the combined detection of NTproBNP/BNP and DE can improve the diagnostic value and help clinical decision.

Nevertheless, there are several limitations regarding this study. First of all, there is noticeable heterogeneity across studies both in terms of the spectrum of the underlying congenital heart disease and the age of the patients. Secondly, two essays used for NTproBNP/BNP measurement and we used cut-off values for PAH diagnosis respectively here. Finally, both invasive and noninvasive measurements were carried out within 72 h in our study; however, PASP can fluctuate widely within a single day due to the variability of pulmonary vascular resistance.

## 5. Conclusion

Our study shows that the Doppler echocardiography combined with NTproBNP/BNP has better diagnostic performance in pulmonary artery hypertension associated with congenital heart disease, especially when DE negative screening in PAH patients.

## Figures and Tables

**Figure 1:** Relationship between PASP estimated by DE and measured by RHC (*r* = 0.4401, *P* < 0.01). DE: Doppler echocardiographic; RHC: right heart catheterization; *r*: correlation coefficient (Pearson); PASP: pulmonary artery systolic pressure.

**Figure 2:** The Bland-Altman plot of PASP estimated by DE and RHC. The bias was 3.2 mmHg, and the 95% limits of agreement were -49.53–55.90 mmHg. PASP: pulmonary artery systolic pressure; DE: Doppler echocardiography; RHC: right heart catheterization.

**Figure 3:** Receiving operator curves using DE and NTproBNP/BNP plasma levels for diagnosis of PAH. (a) The diagnostic performance of DE, NTproBNP/BNP, and DE combined with NTproBNP/BNP for PAH-CHD. (b) The area under the curve (AUC) for the DE was 0.848, for NTproBNP/BNP levels was 0.804, and for the combination of DE and NTproBNP/BNP was 0.857.

**Table 1:** Baseline characteristics and hemodynamics measured by RHC and estimated by DE of the patients.

Male, *n* (%)	18 (28.1%)
Age (mean ± SD, years)	43.8 ± 18.3
ASD, *n* (%)	37 (57.8%)
VSD, *n* (%)	19 (29.7%)
PDA, *n* (%)	8 (12.5%)
PASP measured by RHC (mmHg)	78.1 ± 29.0
PASP estimated by DE (mmHg)	74.9 ± 19.7

ASD: atrial septal defects; VSD: ventricular septal defects; PDA: patent ductus arteriosus; DE: Doppler echocardiography; RHC: right heart catheterization; PASP: pulmonary artery systolic pressure.

**Table 2:** The diagnostic performance of DE and DE combined with NTproBNP/BNP for PAH.

	Ss	Sp	PPV	NPV
DE	98.3%	77.8%	96.6%	87.5%
NTproBNP/BNP	81.4%	87.5%	98.3%	35%
DE+ NTproBNP/BNP	100%	77.8%	96.6%	100%

DE: Doppler echocardiographic; Ss: sensitivity; Sp: specificity; PPV: positive predictive value; NPV: negative predictive value.

## Data Availability

The data used to support the findings of this study are included within the article.
